The article "Effects of Irrational Use of Antibiotics on Intestinal Health of Children with Extraintestinal Infectious Diseases" was retracted in 2023. Reasons: signs of a paper mill; suspected computer-generated content; unreliable results or conclusions; lack of ethics approval or compliance.

# Effects of Irrational Use of Antibiotics on Intestinal Health of Children with Extraintestinal Infectious Diseases

**DOI:** 10.1155/2022/9506490

**Published:** 2022-08-18

**Authors:** Xiaomei Guo, Lifu Sun, Shengjiang Wang, Yan Shen

**Affiliations:** Pharmacy Department, Tongxiang Second People's Hospital, Tongxiang 314511, China

## Abstract

The effects of different antibiotic treatment regimens on intestinal function and flora distribution in children with extraintestinal infectious diseases are explored. A total of 150 cases of extraintestinal infectious diseases admitted to our hospital from January 2021 to January 2022 and 50 healthy subjects during the same period were selected for the study. These 150 children were randomly divided into cephalosporin group, piperacillin group, and combined group and were successively treated with ceftazidime, piperacillin, and two drug combination regimens. The efficacy of the drug, intestinal microflora, intestinal mucosal barrier function, and incidence of antibiotic-associated diarrhea (AAD) were compared among the different groups. The experimental results showed that ceftazidime combined with piperacillin can effectively improve the intestinal health of children with extraintestinal infectious diseases but destroy the microecological environment of intestinal flora, affect the intestinal mucosal barrier function, and increase the risk of AAD.

## 1. Introduction

Extraintestinal infection refers to diarrhea caused by infection of organs outside the digestive tract, in which the skin, lungs, pharynx, and urinary tract are common infection sites, with a high incidence in young, underdeveloped, and weak immunity groups such as neonates [1]. Antimicrobial therapy is the preferred way of treating clinical infectious diseases, but excessive application of antimicrobial drugs can cause intestinal flora disturbance. The distribution of intestinal pathogenic bacteria has significant influence on the function of the intestinal; therefore, in the antimicrobial treatment for intestinal infection diseases, maintaining intestinal flora and improving intestinal barrier function is key to selecting a clinical regimen [2, 3]. Currently, for various combinations of antimicrobial agents that treat intestinal infectious diseases in children, no research has given a unified conclusion. In this study, we used the contrast analysis of antimicrobial agents used alone and in combination to treat intestinal infectious diseases in children, and it provided a new train of thought for subsequent clinical medicine scheme optimization.

The rest of this paper is organized as follows: Section 2 discusses related work, followed by the medication regimen and our proposed methods in Section 3.  Section 4 shows the experimental results, and Section 5 concludes the paper with summary and future research directions.

The article "Effects of Irrational Use of Antibiotics on Intestinal Health of Children with Extraintestinal Infectious Diseases" was retracted in 2023. Reasons: signs of a paper mill; suspected computer-generated content; unreliable results or conclusions; lack of ethics approval or compliance.

## 2. Related Work

Intestinal diseases of exogenous newborns have a recurrent disease history. The most important one is a bacterial infection in the skin, lung, and pharynx, causing symptoms such as diarrhea, with Gram-negative bacteria being the common infection pathogen. Relatively poor immunity of neonates right after birth, premature rupture of membranes, and amniotic fluid contamination can increase the risk of infection, thereby increasing the incidence of extraintestinal infectious diseases [4].

A large number of microbial population resides in the human intestinal tract, with a total of far more than 1 × 10^14^ microbes and with more than 1000 bacterial types, including Proteobacteria, *Bacteroides*, Actinomycota, Firmicutes, and Verrucomicrobia, 90% of which are *Bacteroides* and Firmicutes [5, 6]. Changes in the type and quantity of gastrointestinal flora are a dynamic process, so the stability of intestinal flora microecology under the combined action of the external environment and the body is of great significance to the body's metabolism, immune regulation, absorption, and digestion [7, 8]. Ponziani et al. [9] pointed out that intestinal flora was related to inflammation, and intestinal flora would change significantly after infection, among which bifidobacteria decreased significantly. Chen [10] found that compared with normal infection in patients with abnormal expression of gut bacteria, including bifidobacteria, lactobacillus decreased significantly, while the number of *Escherichia coli* and enterococcus increased significantly, and the results showed that compared with the control group, children of three groups of medication had a significantly lower number of bifidobacteria and lactobacillus probiotics. In addition, the number of probiotics in the combined group significantly increased compared with that in the two groups which used ceftazidime and piperacillin sodium alone, and the number of spoilage bacteria significantly decreased, suggesting that the intestinal flora of patients with extraintestinal infectious diseases would change. Ceftazidime and piperacillin sodium alone or in combination in the treatment for extraintestinal infectious diseases can improve the intestinal flora status of children, while the combined treatment can promote the growth of probiotics and inhibit the proliferation of spoilage bacteria. The reason may be that both ceftazidime and piperacillin sodium can effectively kill spoilage bacteria, thus promoting the growth of intestinal probiotics, reversing the dominant position of the intestinal flora occupied by spoilage bacteria after infection, and enabling the probiotics to have the growth advantage in intestinal flora, thus improving the microenvironment of intestinal flora [11].

The article "Effects of Irrational Use of Antibiotics on Intestinal Health of Children with Extraintestinal Infectious Diseases" was retracted in 2023. Reasons: signs of a paper mill; suspected computer-generated content; unreliable results or conclusions; lack of ethics approval or compliance.

Antibiotics are effective drugs for the treatment of bacterial infections and have a certain impact on the microenvironment of intestinal flora. However, the unreasonable use of antibiotics will increase the resistance of spoilage bacteria and increase the risk of adverse drug reactions while reducing clinical efficacy [12]. This study proved that the combined treatment effect was better than that of cefazolin and piperacillin alone, but there was no statistical significant difference between the groups, and AAD incidence in the combined treatment group was obviously higher than that in the cefazolin and piperacillin groups. The combination of the two drugs can effectively improve the intestinal digestion and provide a curative effect in children with infectious diseases, but greatly increase the risk of adverse reactions such as AAD. The reason for the above results may be that the combination of drugs can effectively inhibit the growth and colonization of intestinal spoilage bacteria, thereby reducing the immune function of spoilage bacteria products and reducing the risk of invasion of other bacteria and pathogens, thus improving the clinical efficacy. However, compared with the single drug treatment, the combined use of the two antibacterial drugs will increase the resistance of pathogenic bacteria in children, and further increase the risk of abdominal distension, diarrhea, and other adverse reactions. Therefore, medication regimens should be formulated according to the individual situation of children to avoid serious adverse drug reactions caused by irrational drug use [13–15].

Disruption of the homeostasis of intestinal flora is the main cause of diarrhea. The abnormal decrease in the number of probiotics in the intestinal tract and the abnormal increase in the number of pathogenic bacteria lead to disturbance of intestinal microecological flora, destruction of the “microbial membrane” barrier, and intestinal mucosal epithelial injury, which leads to intestinal dysfunction diarrhea [16–19]. Intestinal mucosal barrier functions mainly through lactic acid and diamine oxidase (DAO), and serum D-D-lactic acid is one of the glycolysis products inherently present in intestinal bacteria. There is an increase in the level of DAO, and a highly active enzyme present in the villus of cell cytoplasm increases the intestinal mucosal permeability due to damage of intestinal mucosa. There is a change in the function of DAO and D-lactic acid as well as an abnormal rise in circulation. Therefore, D-lactic acid and DAO can be used as sensitive indicators of intestinal mucosal barrier function [13, 20–22]. This study results showed that compared with the control group, D-lactic acid and DAO are significantly higher in children with intestinal infectious diseases. Consistent with the above research and analysis, infection in children with intestinal flora imbalance results in a decrease in small intestine engraftment resistance, overgrowth of small intestinal bacteria, and an increase in secretion of proinflammatory cytokines, thus causing the destruction of microbial barrier and damaging the intestinal mucosa barrier at the same time. Then, D-lactic acid and DAO are highly expressed. The results of this study showed that D-lactic acid and DAO in the combination group were significantly lower than those in the cephalosporin group and piperacillin group, indicating that the combination of drugs could effectively improve the intestinal microflora and thus reduce intestinal mucosal injury. Analyzing its mechanism may help us promote intestinal flora after using the combination of probiotics, which becomes the dominant bacterium group by breeding and by using probiotics supplement, and normal physiological flora, in turn, stimulate bacteria biological barrier formation. At the same time, the probiotics, by serving as a competitive antagonist against bacteria invasion, repair the intestinal flora film on the surface of the barrier and strengthen the defense function of intestinal mucosa barrier against bacterial pathogen. Probiotics can promote intestinal acidification and endotoxin metabolism by secreting a large number of acid substances, thus reducing the damage caused by endotoxin to intestinal mucosa and playing the role of protecting intestinal mucosal barrier and preventing diarrhea [23–26].

The article "Effects of Irrational Use of Antibiotics on Intestinal Health of Children with Extraintestinal Infectious Diseases" was retracted in 2023. Reasons: signs of a paper mill; suspected computer-generated content; unreliable results or conclusions; lack of ethics approval or compliance.

## 3. Medication Regimen and the Proposed Methods

A total of 150 children with extraintestinal infectious diseases treated in our hospital from January 2021 to January 2022 were selected and included in the medication group, and randomly divided into cephalosporin group, piperacillin group, and combined group. The ratio of male to female in the cephalosporin group was 23/27, 35 d to 3 years old, with an average of (1.52 ± 0.53) years old. The male to female ratio in the piperacillin group was 22/28, aged 34 d to 3 years, with an average of (1.54 ± 0.50) years. The male to female ratio in the combined group was 21/29, aged 34 d to 3 years, with an average of (1.51 ± 0.52) years. Inclusion criteria include the following: (1) not taking any antibacterial drugs within one week before participating in the study; (2) informed consent voluntarily signed by the families of the children after clarifying the content and significance of the study; (3) no obvious allergic reaction to antibacterial drugs; (4) diagnosis of extraintestinal infectious by clinical examination; and (5) children under the age of 4. . Exclusion criteria include the following: (1) ceftazidime and piperacillin used in this study having obvious allergic reactions or contraindications; (2) complications with severe organ failure; and (3) incomplete clinical data. In addition, 50 healthy subjects who underwent physical examination at the same period were included in the control group, with a male to female ratio of 24/26, aged 34 d to 3 years old, with an average of (1.52 ± 0.52) years old. There was no statistical difference in the general data of the included subjects (*P* > 0.05), which can be compared effectively.

### 3.1. Medication Regimen

All the subjects in the medication group were given routine treatment after admission, including oxygen inhalation and nutritional support, and the children underwent an antibacterial needle test. If the subjects were found to be allergic to cephalosporin and piperacillin, the treatment was immediately stopped. The piperacillin group was given piperacillin sodium injection (Qilu Pharmaceutical Co., Ltd, Batch No. QL20150102, specification: 1.25 g/piece) as intravenous therapy, 100–150 mg/(kg·d) for 1 week, with an 8 h medication interval.

Children in the cephalosporin group were given ceftazidime injection (Kazakhstan Pharmaceutical Group Pharmaceutical General Factory, Batch No. H20141226, specification: 1.0 mg/piece), with a therapeutic dosage of 30–100 mg/(kg·d), and with an medication interval of ≥8 h, twice a day, for 1 week.

The combination group was given piperacillin sodium injection and ceftazidime injection according to the above two drug regimen. The dosage of piperacillin sodium injection was 30–50 mg/(kg·d), and the dosage of ceftazidime injection was 10–30 mg/(kg·time) for 7 days consecutively, given at an interval of 12 h, twice a day.

### 3.2. Collection and Detection of Intestinal Colony Samples

After treatment, fecal samples of the subjects in the four groups were collected for bacterial culture, and then placed in the K2000 automatic bacterial analyzer (Jilin Keer BioInstrument Co., Ltd) for detection, and the number of intestinal colonies of probiotics such as lactobacillus and bifidobacteria as well as enterococcus and other putrefied bacteria in each group was analyzed.

### 3.3. Detection of Intestinal Mucosal Barrier Function Indicators

DAO and serum D-lactic acid levels were determined by Enzyme-Linked ImmunoSorbent Assay (ELISA).

The article "Effects of Irrational Use of Antibiotics on Intestinal Health of Children with Extraintestinal Infectious Diseases" was retracted in 2023. Reasons: signs of a paper mill; suspected computer-generated content; unreliable results or conclusions; lack of ethics approval or compliance.

### 3.4. Efficacy Evaluation Criteria

The treatment was considered to be efficient if the following indications were observed: complete disappearance of clinical symptoms and significant decrease in the temperature of the children. The treatment was found to be inefficient if the clinical symptoms of the children did not significantly improve or were even worse. The proportion of cured, efficacious, and effective patients was recorded as the total effective rate.

### 3.5. Statistical Methods

The software that effectively processed the data in the study was SPSS 22.0 to test the normality of the measurement data. The normal distribution of the measurement data was presented in the form of ($\bar{x}\pm s$), the *t* test was adopted, *n* (%) was used to represent the count data, and the *x*^2^ test was performed. *P* < 0.05 indicated that the data are statistically significant.

## 4. Experimental Results

### 4.1. Efficacy Comparison

Table 1 shows the comparison of intervention effect indexes in each group. It can be seen from Table 1 that the combined group had a higher total effective rate and shorter cure time than the cephalosporin group and the piperacillin group, but there was no statistical difference between the groups (*P* > 0.05).

### 4.2. Comparison of Changes in Intestinal Flora Quantity

Table 2 shows the comparison of changes in intestinal flora number.  Figure 1 shows the number of intestinal flora in each group. Through the above experimental results, it can be observed that the number of bifidobacteria and lactobacillus in the cephalosporin group, piperacillin group, and combined group decreased compared with the control group and was the lowest in the combined group. The number of *Escherichia coli* and enterococcus in the medication group was higher than that in the control group and was the highest in the combined group, with statistical differences between the groups (*P* < 0.05).

### 4.3. Comparison of Intestinal Mucosal Barrier Function Indicators

Table 3 shows the comparison of intestinal mucosal barrier function indexes.  Figure 2 shows the changes of intestinal mucosal barrier function indexes among groups. It can be observed from Table 3 and Figure 2 that serum D-lactic acid and DAO in the cephalosporin group, piperacillin group, and combined group were higher than those in the control group, and they were the lowest in the combined group. There are statistical differences between the groups (*P* < 0.05).

### 4.4. Comparison of Adverse Reactions

Compared with the cephalosporin group and piperacillin group, the incidence rate of antibiotic-associated diarrhea (AAD) in the combined group was significantly higher, 10.00%, 10.00%, and 28.00%, respectively. There are statistical differences between the groups (*x*^2^ = 5.263, *P*=0.022).

The article "Effects of Irrational Use of Antibiotics on Intestinal Health of Children with Extraintestinal Infectious Diseases" was retracted in 2023. Reasons: signs of a paper mill; suspected computer-generated content; unreliable results or conclusions; lack of ethics approval or compliance.

## 5. Conclusion and Future Work

The effects of different antibiotic treatment regimens on intestinal function and flora distribution in children with extraintestinal infectious diseases are explored. There are still some shortcomings in this study, such as small sample size and few types of antibiotics included, which make the study design incomplete. More antibiotics should be included as observation drugs in the future, and the evaluation of the effect of multiple antibiotics combination should be carried out on the basis of expanding the sample size.

In conclusion, the combined treatment of ceftazidime and piperacillin in children with extraintestinal infectious diseases can effectively improve the clinical efficacy, but will cause intestinal mucosal barrier damage and destroy the stability of intestinal microflora microecological environment, and increase the risk of AAD in children. Therefore, rational medication should be used in the clinical treatment of extraintestinal infectious diseases.

## Figures and Tables

**Figure 1:** Number of intestinal flora in each group.

**Figure 2:** Changes of intestinal mucosal barrier function indexes among the groups.

**Table 1:** Comparison of intervention effect indexes in each group [($\bar{x}\pm s$, %) *n* = 50].

Group	Cure	Excellence	Effective	Invalid	Total effective rate
Cephalosporin group	13 (26.00)	12 (24.00)	15 (30.00)	10 (20.00)	40 (80.00)
Piperacillin group	14 (28.00)	13 (26.00)	14 (28.00)	9 (18.00)	41 (82.00)
Combined group	14 (28.00)	14 (28.00)	16 (32.00)	6 (12.00)	44 (88.00)
*x * ^2^					2.321
*P*					0.324

**Table 2:** Comparison of changes in intestinal flora number ($\bar{x}\pm s$, *n* = 50).

Group	Probiotics (log10^n^/g)		Putrefying bacteria (log10^n^/g)	
	*Bacillus lactis*	Bifidobacterium	*E*. *coli*	Enterococcus
Control group	15.52 ± 1.65	16.61 ± 0.51	4.48 ± 0.22	5.13 ± 0.10
Cephalosporin group	10.52 ± 1.15	12.01 ± 0.41	14.49 ± 0.52	17.83 ± 0.19
Piperacillin group	10.56 ± 1.19	12.06 ± 0.38	14.51 ± 0.57	17.86 ± 0.21
Combined group	12.47 ± 1.21	14.31 ± 0.41	10.32 ± 0.34	13.83 ± 0.14
*F*	14.232	25.343	24.323	24.655
*P*	0.008	<0.001	0.001	0.001

**Table 3:** Comparison of intestinal mucosal barrier function indexes ($\bar{x}\pm s$, *n* = 50).

Group	D-Lactate (ng/ml)	DAO (U/ml)
Control group	0.97 ± 0.16	1.25 ± 0.21
Cephalosporin group	1.87 ± 0.34	2.09 ± 0.40
Piperacillin group	1.82 ± 0.32	2.11 ± 0.37
Combined group	1.47 ± 0.24	1.71 ± 0.32
*F*	22.565	27.564
*P*	0.003	<0.001

## Data Availability

The simulation experiment data used to support the findings of this study are available from the corresponding author upon request.
